The article "Cellular elements for seeing in the dark: voltage-dependent conductances in cockroach photoreceptors" was published in 2012. Journal: BMC Neurosci.

# Cellular elements for seeing in the dark: voltage-dependent conductances in cockroach photoreceptors

**DOI:** 10.1186/1471-2202-13-93

**Published:** 2012-08-06

**Authors:** Iikka Salmela, Esa-Ville Immonen, Roman Frolov, Stephan Krause, Yani Krause, Mikko Vähäsöyrinki, Matti Weckström

**Affiliations:** 1 Department of Physics, University of Oulu, Oulu, Finland

**Keywords:** Potassium channel, Sensory neuron, Photoreceptor

## Abstract

**Background:**

The importance of voltage-dependent conductances in sensory information processing is well-established in insect photoreceptors. Here we present the characterization of electrical properties in photoreceptors of the cockroach (*Periplaneta americana*), a nocturnal insect with a visual system adapted for dim light.

**Results:**

Whole-cell patch-clamped photoreceptors had high capacitances and input resistances, indicating large photosensitive rhabdomeres suitable for efficient photon capture and amplification of small photocurrents at low light levels. Two voltage-dependent potassium conductances were found in the photoreceptors: a delayed rectifier type (KDR) and a fast transient inactivating type (KA). Activation of KDR occurred during physiological voltage responses induced by light stimulation, whereas KA was nearly fully inactivated already at the dark resting potential. In addition, hyperpolarization of photoreceptors activated a small-amplitude inward-rectifying (IR) current mediated at least partially by chloride. Computer simulations showed that KDR shapes light responses by opposing the light-induced depolarization and speeding up the membrane time constant, whereas KA and IR have a negligible role in the majority of cells. However, larger KA conductances were found in smaller and rapidly adapting photoreceptors, where KA could have a functional role.

**Conclusions:**

The relative expression of KA and KDR in cockroach photoreceptors was opposite to the previously hypothesized framework for dark-active insects, necessitating further comparative work on the conductances. In general, the varying deployment of stereotypical K^+^ conductances in insect photoreceptors highlights their functional flexibility in neural coding.

## Background

In sensory cells, voltage-gated ion channels shape the voltage responses arising from currents generated in sensory transduction processes. The biophysical properties of the channels allow them to change the electrical properties of the membrane in a voltage- and time-dependent manner, which in graded potential neurons and sensory cells lead to amplification of relevant and attenuation of irrelevant signals. In this way ion channels can effectively regulate the membrane according to the requirements set by the input (e.g. the transduction currents) and, in general, the sensory ecology of the animal [1]. Expressing a suitable composition of specific channel types enables tuning of the information coding performance versus the metabolic cost of voltage signalling [2-4].

The article "Cellular elements for seeing in the dark: voltage-dependent conductances in cockroach photoreceptors" was published in 2012. Journal: BMC Neurosci.

Photoreceptors form a well-established model system for examining the specific molecular mechanisms involved in processing sensory information that is carried by graded voltage signals in both vertebrates [5-7] and insects [8,9]. In flies, photoreceptors of fast-flying diurnal species possess a distinctively different set of voltage-gated potassium channels (Kv-channels) than those of slower and crepuscular species [10,11]. Photoreceptors of diurnal flies rely on non- or slowly inactivating delayed rectifier (DR) channels, whereas nocturnal or crepuscular flies express mainly inactivating Kv channels [10-12]. The DR channels in the dawn and dusk active fruit fly (*Drosophila melanogaster*) are responsible for attenuating the light-dependent depolarization and speeding up the membrane filter at higher light levels [13-15], whereas the rapidly inactivating transient A-type channels dynamically shape the transient signals to enable full use of the available voltage range [3]. This allows *Drosophila* photoreceptors to extract information efficiently from the dynamic light stimuli and to encode it into voltage responses of limited amplitude and speed without excessive metabolic costs [3,4,13].

Cockroaches are mainly dark-active, but can also aggregate in daylight [16]. While they rely heavily on mechano- and chemosensory systems when gathering information about their surroundings [17,18], vision also appears to play a significant role in their behaviour [19-21]. The importance of vision can also be inferred from the large compound eyes (over 3000 ommatidia per eye [22]) that have been maintained through evolution for hundreds of millions of years, despite the associated metabolic cost [23,24]. Therefore, cockroaches form an interesting model system for studying mechanisms of vision under dark conditions when the rate of photons arriving in the eye is small.

While several studies on vision of nocturnal insects have been published [25], a detailed characterization of the biophysical properties of photoreceptors has not been previously performed in any dark-active insect. Our earlier investigations have revealed several peculiar features of the cockroach photoreceptors, e.g. exceptional action potential coding in the axons [26] and nearly randomly varying functional properties [27], both of which were interpreted as adaptations to nocturnal vision. In this study, we have characterized the biophysical properties of the voltage-dependent conductances in the somata of dissociated cockroach photoreceptors using the patch-clamp method. Mathematical modelling was performed to circumvent experimental limitations in monitoring the simultaneous interplay of different conductances during voltage responses to light. Relative contributions of the characterized conductances in shaping physiologically relevant signals were calculated and discussed with respect to the previously proposed hypothesis for the roles of different types of Kv-channels in photoreceptors of insect species with varying visual ecology.

The article "Cellular elements for seeing in the dark: voltage-dependent conductances in cockroach photoreceptors" was published in 2012. Journal: BMC Neurosci.

## Methods

### Electrophysiology

All experiments were performed using adult male cockroaches *Periplaneta americana* obtained from Blades Biological Ltd (Edenbridge, Kent, UK). The animals were kept at 25°C in a 12 h day-night rhythm. The ommatidia dissociation procedure was similar as described previously for *Drosophila*[15]. In brief, after decapitation and removal of antennae, eyes were cut off with a sharp razor blade. Retinas were scooped out and cut into several pieces. The retinal fragments were then incubated for 8-10 min in extracellular solution supplemented with 0.2 mg/ml collagenase type 2 (Worthington Biochemical Corp., Lakewood, NJ USA) and 0.2 mg/ml Pankreatin (Sigma-Aldrich) followed by gentle trituration with systematically varying the tips of the trituration pipettes, until ommatidia started to fall off. Separate ommatidia were allowed to settle in the recording chamber on the stage of an inverted microscope (Axiovert 35 M, Zeiss, Germany). The preparation and the recordings were done at room temperature (20-23°C).

Patch-clamp recordings were performed using an Axopatch 1-D amplifier (Molecular Devices, USA) and pCLAMP 9 software (Molecular Devices, USA). Patch microelectrodes were made from borosilicate glass (Harvard Apparatus Ltd, UK) using a P-87 electrode puller (Sutter Instrument Company, Ca, USA) and had resistances between 5 and 15 MΩ. Access resistances were monitored throughout the experiment and after 80-90% compensation they were typically well below 10 MΩ. Voltage errors caused by access resistance were corrected offline for currents larger than ± 200 pA.

The standard bath solution contained (in mM): 120 NaCl, 5 KCl, 4 MgCl_2_, 1.5 CaCl_2_, 10 N-Tris-(hydroxymethyl)-methyl-2-amino-ethanesulfoncic acid (TES), 25 L-proline and 5 β-alanine, pH 7.15 (NaOH). For experiments involving K^+^ gradients we prepared a high K^+^ concentration bath solution containing (in mM): 120 NaCl, 50 KCl, 4 MgCl_2_, 1.5 CaCl_2_, 10 TES, pH was adjusted to 7.15 (NaOH). The standard and high K^+^ bath solutions were mixed in relevant proportions to receive K^+^ concentrations of 5, 15, 25 and 50 mM.

The article "Cellular elements for seeing in the dark: voltage-dependent conductances in cockroach photoreceptors" was published in 2012. Journal: BMC Neurosci.

Electrode solutions contained (in mM) either 140 K-gluconate (referred to as Cl-free) or 140 KCl (referred to as Cl-containing) together with 10 TES, 2 MgCl_2_, 4 Mg-ATP, 0.4 Na-GTP and 1 NAD, pH was adjusted to 7.15 (KOH). Properties of K^+^ currents were studied using Cl-free solutions, while experiments involving the study of the inward current or voltage and current responses to light stimuli were performed with the Cl-containing electrode solution. All chemicals were purchased from Sigma-Aldrich.

All recordings were done from green-sensitive photoreceptors, identified by their response to stimulation with a green LED (525 nm). Whole-cell input resistances, capacitances and access resistances were determined offline from voltage clamp experiments with a hyperpolarizing voltage step, using the test pulse method described in pCLAMP 9 manual.

Light responses were recorded by stimulating the photoreceptors with an LED through the fluorescence port of the microscope. LED intensity was controlled with a voltage-current converter and the acquisition hardware and software. Voltage light responses were recorded in the amplifier’s current clamp mode (I = 0) and the light-induced currents (LIC) in the voltage-clamp mode, with a holding potential of 74 mV. Light stimuli were either pulses or a dynamic waveform taken from the van Hateren naturalistic time series intensity (NTSI) database [28].

### Data analysis and mathematical modeling

Data were analyzed using OriginPro 8.5 (Originlab, US). Conductances were calculated from currents recorded in different holding potentials *V* as *g* = *I*/(*V* -*E*_*rev*_), where *I* is the current and *E*_*rev*_ is the reversal potential. The voltage values presented in the text were corrected for the liquid junction potential (LJP) unless stated otherwise.

Kinetic parameters of gating of K^+^ currents, recordings of light-induced current in response to a 10 s naturalistic light contrast sequence [28], and the corresponding voltage responses obtained from patch clamp experiments were used in a Hodgkin-Huxley type mathematical model implemented in Matlab (Mathworks, USA). The model was then used to study the relative contribution of ionic conductances during simulated light responses. The model is described in detail in the Appendix.

## Results

### General properties of cockroach photoreceptors

Isolated cockroach ommatidia were between 100 and 150 μm long and ca. 30 μm wide (Figure 1A) and normally did not contain the photoreceptor axons. In patch clamp experiments, the seal resistance was typically greater than 10 GΩ and the whole-cell input resistance (*R*_*in*_) in darkness varied between 200 MΩ and 10 GΩ (*R*_*in*_ = 1.6 ± 2.4 GΩ, n = 32). The *R*_*in*_ values were larger than the previous estimates from *in vivo* intracellular recordings [26,27], possibly because of the absence of a membrane leak due to membrane piercing with a sharp glass microelectrode [29]. Whole-cell membrane capacitance was measured as a proxy for the membrane area and cell size, which are known to vary within single ommatidia [30]. The capacitances ranged from 100 to 800 pF (Figure 1B) and did not follow a normal distribution, which may reflect different photoreceptor size groups in the ommatidia [30]. We cannot rule out the possibility that some recordings with the largest capacitances could contain more than one cell. However, such occurrences have not been reported before with insect photoreceptors in patch clamp, although in intracellular recordings it is possible [31].

The article "Cellular elements for seeing in the dark: voltage-dependent conductances in cockroach photoreceptors" was published in 2012. Journal: BMC Neurosci.

**Figure 1:** **General features of isolated photoreceptors. A**) Isolated ommatidia of *Periplaneta americana. * Single photoreceptors cluster with their fused rhabdom concentrically around the longitudinal axis of the ommatidium. The rhabdom can be recognized as a dark central structure. Lenses at the distal end (top) and axons at the proximal end (bottom) are ripped off during isolation. Note the pigmentation of the ommatidia. **B**) Whole-cell capacitances of green-sensitive photoreceptor cells (n = 45). **C**) Current responses to 1 ms dim light flash stimuli containing less than 1 photon on average showed both single photon absorptions (+) and failures (-). The variability of response latency and amplitude reflects the random properties of phototransduction. The holding potential in voltage clamp mode was -77 mV. **D**) Voltage responses (top) and corresponding light-induced-currents (middle) to a 10 s long naturalistic light intensity series (bottom) recorded in whole-cell patch clamp. Relative intensities were 1 (gray traces) and 10 (black trace). **E**) In whole-cell current clamp recordings, voltage responses (top) to current injections (bottom) exhibited both inward- and outward rectification, indicating the presence of voltage-dependent conductances. The small-amplitude depolarizations are single photon responses to ambient light.

Photoreceptors in isolated ommatidia were functionally robust, with light responses occasionally recorded for over one hour of continuous light stimulation. Figure 1C shows quantum bumps, which are current responses to single-photon stimulation. Quantum bumps could be recorded from all the cells used in the analyses and their presence was used as an indicator of photoreceptor health. Examples of macroscopic current and voltage responses elicited by a 10 s naturalistic light stimulus [28] are shown in Figure 1D. Hyperpolarizing and depolarizing current steps in darkness produced voltage responses characterized by a slow passive membrane time constant (170 ms for the -50 pA trace in Figure 1E). The rectification, i.e. the nonlinear, asymmetric behaviour of voltage in response to depolarizing and hyperpolarizing current injections (Figure 1E), demonstrated the presence of voltage-dependent conductances, which were then studied further.

The article "Cellular elements for seeing in the dark: voltage-dependent conductances in cockroach photoreceptors" was published in 2012. Journal: BMC Neurosci.

### Voltage-activated K^+^ (Kv) currents

Voltage clamp experiments revealed a voltage-activated outward current (Figure 2) responsible for the rectification observed at depolarized voltages in current clamp recordings (Figure 1E). Kinetics and amplitude of the outward current varied from cell to cell (Figure 2A-B). In approximately half of the photoreceptors, the current clearly consisted of two components: a fast-activating transient current and a slow-activating sustained current (Figure 2B). The sustained current showed no inactivation during prolonged voltage pulses (Figure 2C).

**Figure 2:** **Outward currents in photoreceptors.** Voltage-clamp recordings revealed of voltage-dependent outward currents that could be activated with depolarization the cell. The outward current consisted of at least two components, the amount of which varied between cells. **A**) A photoreceptor with large transient current **B**) A photoreceptor with both transient and sustained currents **C**) The sustained current did not inactivate during a 10 s long voltage clamp. Voltage was clamped from -47 mV to +3 mV with 10 mV intervals after a -117 mV prepulse. **D**) Depolarizing pulses from -57 to +3 mV given after a hyperpolarizing -117 mV pre-pulse elicited both a sustained and a transient outward current **E**) Positive prepulse inactivated the transient component, and subsequent depolarization activated only the sustained current. **F**) The transient current could be isolated by subtraction of the currents from protocols in D) and E). The scale bar applies for panels D, E, and F.

The transient current displayed voltage-dependent inactivation whereas the sustained current did not, thus allowing separation of the two current components by voltage clamp protocols. Depolarizing pulses given after a prepulse of -117 mV activated both the transient and the sustained current (Figure 2D). Depolarizing pulses following a -57 mV prepulse evoked only the sustained current (Figure 2E), due to the inactivation of the transient current by the pre-pulse. The current obtained by subtraction of the currents evoked by the two protocols was taken as the transient current (Figure 2F). The voltage-dependences of the sustained and the transient current resembled delayed-rectifier and A-type Kv currents, respectively, both of which are commonly found in neurons [32,33], including insect photoreceptors [3,11-13,15].

The article "Cellular elements for seeing in the dark: voltage-dependent conductances in cockroach photoreceptors" was published in 2012. Journal: BMC Neurosci.

The sustained current’s identity and selectivity was examined with tail currents recorded under different external potassium concentrations (Figure 3). The fitted Nernst slope was 52 ± 4 mV/mM (mean ± SE), close to the theoretical value of 58 mV/mM for potassium with the solutions used. Under standard K^+^ concentrations ([K]_in_/K]_out_ = 5 mM/140 mM) the reversal potential of the current was -68 ± 5 mV (mean ± SD, n = 17). Theoretical Nernst potential for potassium was -84 mV, implying that the measured conductance was not entirely potassium-specific under multi-ionic conditions. The reversal potential was similar for chloride-containing and chloride-free solutions (see Methods for a description of solutions). Because of the overlap with the sustained current, the transient current’s reversal potential could not be measured reliably but was assumed to be the same as for the non-inactivating current, i.e. -68 mV, based on the close resemblance of both to K^+^ currents in insects [33]. The similarity of the voltage-dependent behaviour of the currents to previous findings in insects (Figure 2D-F) and the Nernst slope of the sustained current’s reversal potential (following K^+^ concentration and thus indicating a mainly K^+^ permeant channels; Figure 3) indicate that the currents are generated by voltage-dependent potassium (Kv) channels. Based on their similarities to delayed-rectifier and A-type Kv currents, the non-inactivating sustained current will be referred as KDR and the inactivating transient current as KA in the following.

**Figure 3:** **Reversal potential of the sustained current followed the Nernst slope for potassium.** The reversal potential was measured from tail currents with varying external K^+^ concentrations (inset), resulting in E_rev_ = -68 mV under the standard 5 mM concentration (n = 17 (5 mM), 6 (15 and 50 mM) or 5 (25 mM), data are mean ± SD). The fitted Nernst slope (solid line) was 52 mV/mM and the theoretical Nernst slope (dashed line) for potassium was 58 mV/mM. Theoretical *E*_*rev*_ with 5 mM [K^+^]_out_ was -84 mV.

KDR was isolated by giving voltage pulses from -47 to +23 mV in 10 mV steps after a -57 mV prepulse that inactivated the KA conductance (Figure 2E). Conductances were calculated from the steady-state currents and fitted with first order Boltzmann function *g*(*V*) = *g*_*max*_/(1 + exp((*V*_*50*_ - *V*)/*slope*)), corresponding to 1^st^ order kinetics for the activation. The resulting half-activation voltage (*V*_*50*_) was -31 ± 9 mV with *slope* factor of 12.0 ± 2.0 mV, and the maximum conductance (*g*_*max*_) was 78 ± 22 nS (mean ± SD, n = 6), ranging between 40 and 90 nS. A normalized KDR activation profile is shown in Figure 4A (black squares and curve). Activation and deactivation kinetics were determined from single-exponential fits to activating currents or deactivating tail currents. At physiologically relevant voltages from -70 to -10 mV, KDR activation time constants fell between 20 and 11 ms (Figure 4B black squares).

The article "Cellular elements for seeing in the dark: voltage-dependent conductances in cockroach photoreceptors" was published in 2012. Journal: BMC Neurosci.

**Figure 4:** **Voltage-dependent properties of the Kv currents. A**) Steady state activation and inactivation properties of the Kv currents (all data are mean ± SD). Black squares represent activation of the sustained KDR current (n = 6); gray symbols represent transient KA current’s activation (circles, n = 5) and inactivation (triangles, n = 4). The curves are the corresponding Boltzmann fits: KDR activation is a 1^st^ order Boltzmann with V_50_ = -31 mV and slope = 12 mV. KA activation is a 2^nd^ order Boltzmann with *V*_*50*_ = -43 mV and slope = 8.4 mV. KA inactivation is a 1^st^ order Boltzmann with *V*_*50*_ = -85 mV and slope = -11 mV. **B**) Activation time constants of KDR (black squares, n = 8 to 14) and KA (gray circles, n = 5). KDR activation time constant was fitted with a bell-function τ_KDR_ = 1/(4·exp(-43*V) + 156·exp(43*V)) s, where V is voltage in volts. KA activation time constant was nearly voltage-independent and was thus set to constant 1.5 ms for the simulations. **C**) Time constant of the KA inactivation (n = 3 to 7). Bell function is *τ*_*KA*_ = 1/(341 ·exp(44·*V*) +0.211·exp(-44·*V*)) s, where *V* is voltage in volts. Inset: the inactivation recovery protocol used for voltages below -80 mV.

Voltage-dependence of KA activation was determined with the voltage clamp subtraction protocol (Figure 2D-E). Peak conductances were then calculated from the peak currents and fitted with a 2^nd^ order Boltzmann function *g*(*V*) = *g*_*max*_/(1 + *exp*((*V*_50_ - *V*)/*slope*))^2^ , corresponding to 2^nd^ order activation kinetics for the KA channels. The half-activation potential for the 2^nd^ order Boltzmann was -43 ± 4 mV with slope of 8.4 ± 1.6 mV (mean ± SD, n = 5). The normalized activation profile for KA is shown in Figure 4A (gray circles and curve; note that because the activation function is of the 2^nd^ order, the V_50_ value in the equation did not here translate into the 50% value of the activation). Voltage-dependence of KA inactivation was determined from the peak currents, elicited by a -7 mV command pulse following an inactivating prepulse. A first order Boltzmann fit to the peak currents gave a half-inactivation potential of -85 ± 1 mV and a slope factor of -11.3 ± 2.9 mV (Figure 4A, gray triangles and curve, mean ± SD, n = 4). Activation and inactivation time constants were fitted to the subtraction protocol currents with a pulse function, *I* = *I*_max_·(1 -exp(-*t*/*τ*_act_)^2^·exp(-*t*/*τ*_inact_)). Due to the large capacitive transient in whole-cell voltage clamp recordings, the rapid activation kinetics of KA could not be acquired reliably. Nonetheless, the activation time constant was fast at around 1-2 ms (Figure 4B, gray circles, mean ± SD, n = 5), and thus several fold faster than activation of KDR. KA inactivation time constants were obtained from either subtraction protocol currents or from the inactivation recovery (Figure 4C, inset). KA inactivation time constants (Figure 4C) ranged between 50 and 5 ms at physiologically relevant voltages (-70 to -10 mV). The maximum KA conductance was 36 ± 29 nS (mean ± SD, n = 5) and ranged between 11 and 79 nS.

The article "Cellular elements for seeing in the dark: voltage-dependent conductances in cockroach photoreceptors" was published in 2012. Journal: BMC Neurosci.

### Kv currents and photoreceptor size

The whole-cell capacitance results from the photoreceptor membrane, which includes the folded microvillar membrane of the rhabdomere and the unfolded membrane of the soma. The differences in measured capacitances (Figure 1B) could thus reflect the variable size of photoreceptors, or alternatively the sizes of their rhabdomeres or somas, or both. If the differences in capacitance were produced by rhabdomere or soma size variation, there should be other differences as well.

To test if the measured capacitances were linked to other photoreceptor properties, we looked at Kv conductances and voltage light responses recorded in the same cells. Kv currents were elicited by a -4 mV voltage step given after a hyperpolarizing inactivation removal pulse. KDR steady-state and KA peak conductances were then calculated from the currents after series resistance correction. Larger KA conductances were found in small cells, whereas no KA conductance could be observed in large cells (Figure 5A). However, the capacitive transient arising from the whole-cell capacitance and access resistance might partly conceal the transient KA current in the cells with large capacitance. KDR conductances were found in all cells, and conductance values showed a positive trend with increasing capacitance (Figure 5B), and KDR conductance density was 0.14 ± 0.06 nS/pF (mean ± SD, n = 23). Voltage responses to a saturating 10 s long light pulse were recorded from the same photoreceptors. The depolarization at the end of the response was taken as a measure of light-induced voltage change that is the result of the interplay between the depolarizing light-induced current and the hyperpolarizing Kv currents that are activated by the depolarization. Light-induced steady-state depolarization was smaller in cells with lower than those with higher capacitances (Figure 5C) and the relationship between the depolarization whole-cell capacitance resembled the variability of light responses as reported by Heimonen et al. (2006). This suggests that the variability reported earlier is related to cell size, possibly due to fewer or more numerous microvilli in the smaller or larger rhabdomeres and, consequently,a smaller or larger amount of transducing channels.

The article "Cellular elements for seeing in the dark: voltage-dependent conductances in cockroach photoreceptors" was published in 2012. Journal: BMC Neurosci.

**Figure 5:** **Small cells have large KA conductances and small depolarization in response to light. A**) KA and **B**) KDR conductances versus the whole-cell capacitances (n = 23). Conductances were calculated from the currents elicited by a voltage jump to -4 mV from -104 mV **C**) The light-induced steady-state depolarization was smaller in cells with lower whole-cell capacitances.

### Pharmacology of Kv channels

Pharmacological properties of Kv currents were tested with a number of Kv channel blockers in whole-cell voltage clamp (Figure 6A-D). 4-aminopyridine (4-AP) typically blocks A-type Kv currents at high micro- to millimolar concentrations [34]. Application of 1 mM 4-AP in the extracellular solution inhibited the transient KA current, but had no effect on the KDR current (Figure 6A). Tetraethylammonium (TEA), a common blocker of delayed rectifier Kv currents, inhibited the non-inactivating KDR only partially at a high concentration of 50 mM (Figure 6B). Quinidine, a non-specific blocker of various Kv currents in insect neurons [15,34], inhibited the transient KA current at 1 mM extracellular concentration (Figure 6C) and the slow-activating KDR (Figure 6D) with half-maximum inhibitory concentration of *IC*_50_ = 32 ± 3 μM and Hill coefficient of 0.97 ± 0.08 (mean ± SE). Although quinidine inhibited the KDR current well, it had other effects, possibly mediated by interference with the light-gated channels or their activation; thus using it during light responses produced inconclusive results and was not investigated further. Application of 100 nM α-dendrotoxin, a potent blocker of Shaker A-type Kv channels [35], did not block KA or KDR (data not shown).

**Figure 6:** **Pharmacological properties of the Kv currents.** Kv currents were elicited with a positive command potential, given after a negative inactivation-removal prepulse. Black traces are controls; gray traces are currents recorded after drug application. **A**) 1 mM 4-AP suppressed the transient KA component. **B**) 50 mM TEA blocked KDR partially. **C**) 1 mM quinidine blocked both KDR and KA. **D**) Concentration dependence of the quinidine block for the KDR (mean ± SD, n = 3 to 5). The fitted curve is a logistical function 1/(1 + ([quin]/*IC*_50_)^*p*^), with half-inhibition concentration *IC*_50_ = 32 ± 3 μM and Hill slope *p* = 0.97 ± 0.08 (mean ± SE).

The article "Cellular elements for seeing in the dark: voltage-dependent conductances in cockroach photoreceptors" was published in 2012. Journal: BMC Neurosci.

### Hyperpolarization-activated inward-rectifying (IR) current

In the Cl-containing bath solution the current clamp recordings exhibited an inwardly-rectifying response to negative current injections (Figure 1E). In the whole-cell voltage-clamp experiments under similar ionic conditions, hyperpolarization of the photoreceptors activated a small inward current (IR, Figure 7A). Increasing the extracellular K^+^ concentration from 5 mM to 20 mM had no effect on the IR current (Figure 7B), indicating that it is neither carried nor modulated by potassium. Substituting the extracellular NaCl with Na-gluconate reduced the IR current amplitude (Figure 7C). The voltage-dependence of the current and the Na-gluconate effect were similar to the CLC-2 channels [36], suggesting chloride as the main current carrier. Because the activation of this current took place in a negative voltage regime compared to the dark resting potential, it was not investigated further here.

**Figure 7:** **Hyperpolarization-activated inward rectifying (IR) current. A**) Hyperpolarizing voltage clamps from -74 mV to -124 mV elicited a small-amplitude IR current that activated slowly and showed no inactivation. The sharp transients at the end of the clamp currents are capacitive transients. **B**) The IR current was insensitive to changes in the external potassium concentration, ruling out potassium as the current carrier. Black circles with [K]_o_ = 5 mM, white squares [K]_o_ = 20 mM (mean ± SEM, n = 4). **C**) Replacing the NaCl in the bath with Na-gluconate reduced the IR current, indicating that the IR current is carried at least partly by chloride. Black circles are controls with NaCl, white squares are substitution experiments with Na-gluconate (mean ± SEM, n = 4).

### Roles of K^+^ conductances in light responses

Responses to 10 s naturalistic light intensity series were recorded in both voltage and current clamp modes (Figure 1D). Recorded light currents were then used for estimation of the light-induced conductance required for the light response in simulations. The light-induced current (LIC) is determined by the light-induced conductance and its driving force (voltage difference between the membrane potential and the LIC reversal potential). Thus, although possible to determine in voltage clamp, it was not possible to measure the actual LIC driving the photoreceptor’s voltage response, when recording in the current clamp mode when the voltage is varying freely. With the model, however, we could indirectly estimate the currents contributing to the voltage responses to moderate intensity light stimulations, based on the experimentally determined light-induced and voltage-gated conductances [13,37].

The article "Cellular elements for seeing in the dark: voltage-dependent conductances in cockroach photoreceptors" was published in 2012. Journal: BMC Neurosci.

To determine the roles of KDR and KA during light responses, a Hodgkin-Huxley type model of a cockroach photoreceptor was implemented following similar approach as previously described in *Drosophila*[3]. The model was based on the experimentally determined light-induced conductance (Figure 1D), the voltage- and time-dependent properties of KA and KDR (Figure 4), and the values of the resting potential, the capacitance and the input resistance. Simulated voltage clamps (Appendix, Figure 8) and light responses to a 10 s naturalistic contrast stimulus (Figure 9A, c.f. Figure 1D) behaved similarly to the experiments, and thus the various currents underlying the voltage responses could be estimated with the model. During the simulated light responses KDR activated strongly, producing currents up to 1 nA (Figure 9B). Conversely, KA currents during the light responses were small and the maximal KA current during the initial voltage transient was only ca. 40 pA (Figure 9C). The strong inactivation at physiological voltages kept KA currents very small throughout the simulations. As a test of the significance of the KDR, its partial removal from the model down to 10% of the mean experimentally determined conductance values increased the depolarization level of the light responses (Figure 10A). Conversely, increasing the KDR conductance up to 10-fold decreased the amplitude and speeded up the voltage response (Figure 10A). Varying the KA maximum conductance from zero to ten-fold from the experimentally determined value had no visible effect on the simulated voltage responses (Figure 10B). Similarly, no effect was found when other steady-state KA parameters were varied within their minimum/maximum experimental ranges, i.e. *V*_*50*_ of activation (-43 to -40 mV) and inactivation (-88 to -84 mV) and the slopes of activation (6.2 to 10.5 mV) and inactivation (-14.3 to -8.5 mV). The possible influence of the dark resting potential on these results was checked by running simulations using resting potentials ranging from -80 to -50 mV. With more hyperpolarized resting potentials the initial KA transients became larger but soon after the onset of the light stimulation the KA quickly inactivated to very low levels, similar to the standard simulation conditions. The overlap between the KA steady-state activation and inactivation (Figure 4D) indicated that the channel is partially activated already at dark resting potential at ca. -60 mV, although the conductance is small (ca. 0.08 nS). Since the graded voltage changes were slow compared to the kinetics of KA, inactivation always dominated and KA thus remained mostly inactivated after the initial transient.

The article "Cellular elements for seeing in the dark: voltage-dependent conductances in cockroach photoreceptors" was published in 2012. Journal: BMC Neurosci.

**Figure 8:** **Validation of voltage-dependent properties in the simulations.** Voltage clamp simulations with the model (left column) resulted in similar current responses as in experiments (right column, c.f. Figure 2D-F in Results). The insets on the left show the voltage protocols used. **A**) The current elicited from voltage jump from -117 mV prepulse up to + 3 mV. **B**) The current elicited by voltage jump from -57 mV prepulse up to +3 mV. **C**) The subtraction current A -B.

**Figure 9:** **Simulated light responses and underlying Kv currents. A**) Voltage responses to the naturalistic light stimulus were simulated with the model (Appendix), using the light-induced conductances calculated from the light-induced currents recorded in voltage clamp (Figure 1D) as input. Relative stimulus intensities were 1 (black) and 10 (grey). **B**) KDR current was activated already at rest and increased further during the light-induced depolarization. **C**) KA currents before and during the light response were small.

**Figure 10:** **Effect of varying the maximum conductances of the KDR and KA in the simulations. A**) Light responses were simulated with 10% (top trace), 100% (gray trace), 200% and 1000% (lowest traces) of the experimentally determined mean KDR maximum conductance. **B**) Modifying the maximal KA conductance had no effect on the simulated light response. The responses were simulated with 0%, 100%, 200% and 1000% KA conductances relative to the standard simulation value of 60 nS. Due to minimal differences in the responses the traces overlap.

## Discussion

Photoreceptors can be used as model systems for signal processing, involving input signals in the form of light-gated current, modulation of the resulting voltage signals by voltage-dependent channels, and output by synaptic transmission to interneurons [7]. Nocturnal or crepuscular insects such as the cockroach have to cope with dim environments, where the reliability of visual information decreases due to the stochastic nature of photon arrival and relatively large transduction noise [38]. We have for the first time characterized in detail the electrical membrane properties in photoreceptors of an insect adapted to dark, the cockroach *Periplaneta americana*.

Several anatomical and physiological strategies for improving dim light vision exist in the insect visual systems. Compound eye optics, photoreceptor properties and the later neural processes can be optimized for efficient light capture and signal transmission [25]. At the photoreceptor level, common strategies used by nocturnal arthropods include temporal summation by the low-pass properties of phototransduction and the photo-insensitive membrane, large-amplitude single photon responses and a large rhabdomere that increases the photon catch [39,40]. Spatial summation of signals from several photoreceptors in the 2^nd^ order neurons of the Lamina can further improve vision under conditions where the number of photons is very small [41-43]. A conclusion that can be made from these studies is that, when only a small number of photons are absorbed by the photoreceptors, sufficient visual information is acquired through sacrificing either spatial or temporal resolution, or both. Our new results show how the voltage-dependent channels fit into this big picture in the cockroach photoreceptors. Both the experimental approach, patch-clamping of the photoreceptors in the isolated ommatidia, and the theoretical approach, mathematical modelling, are used to gain mechanistic understanding. Interestingly, our results show that the Kv channel composition in the cockroach photoreceptors does not follow the pattern found previously in the Diptera [10,11].

The article "Cellular elements for seeing in the dark: voltage-dependent conductances in cockroach photoreceptors" was published in 2012. Journal: BMC Neurosci.

As can be expected, temporal integration in the cockroach photoreceptors is clearly one of the main visual adaptations for life in the dark [27]. It limits coding to the relatively slow visual signals compared to the fast-flying diurnal flies, whose photoreceptors respond to much higher stimulus frequencies [44,45]. In cockroach photoreceptors low-pass filtering arises from the slow phototransduction (Figure 1C-D) and the electrical properties of the membrane (Figure 1E), manifested in the large whole-cell resistance and capacitance. The capacitance ensues from the rhabdomere’s large microvillar area that increases the photon capture efficiency of the cells [46]. The high resistance in the dark and at rest combined with the large capacitance yields a slow time-constant: ca. 60 ms with typical membrane capacitance of 400 pF and resistance of 150 MΩ at -60 mV. This corresponds to a temporal low-pass filter with a cut-off frequency of ca. 3 Hz. For comparison, in dark-adapted photoreceptors of the diurnal blowfly *Calliphora vicina*, membrane resistance and time constant are 32 MΩ and 4 ms, resulting in a corner frequency of 25 Hz, which in light-adaptation is nearly tripled to 72 Hz [12]. In cockroach photoreceptors the high input resistance near the resting potential amplifies single photon responses, enabling large amplitude voltage bumps.

The article "Cellular elements for seeing in the dark: voltage-dependent conductances in cockroach photoreceptors" was published in 2012. Journal: BMC Neurosci.

During light responses the membrane gain and speed are strongly modulated by voltage-gated channels. The dark- and day-active Dipteran fly species possess varying Kv channel compositions dominated by either A-type or DR channels, respectively [10,11]. This is considered to result from the optimization between the need for faster vision and the subsequent increase in the metabolic costs [2,4]. Moreover, some insects that are active during both day and night demonstrate circadian changes in the Kv channels, with transient currents expressed at the night and sustained currents during the day [47,48]. It was therefore surprising that the dominant Kv current in the nocturnal cockroach was the noninactivating KDR (Figure 2).

Our results show that the conductances activated with the depolarization are relatively specific for K^+^, and thus it is plausible that they are created by the Kv-channels (Figure 3). The voltage-activated currents could be separated into two components, the sustained non-inactivating KDR and the transient inactivating current KA (Figure 4. and the Appendix). Although both KDR and KA showed some of the typical characteristics of previously described insect Kv-channels, most importantly the voltage-dependence of activation and inactivation and the sensitivity to various Kv blockers (Figure 6; compare to channels in [33].), the molecular identities of the channels remain unknown. However, the insensitivity of KA to the *Drosophila* Shaker blocker αDTX suggests that KA is not coded by the Shaker gene. KDR was activated already at the -60 mV resting potential in dark, contributing almost 90% of total membrane conductance. Therefore KDR participates in shaping even the smallest light responses, the quantum bumps, and may be required to prevent or attenuate saturation with transient increases of light. Simulations showed that similarly to the sustained Kv currents in the photoreceptors of other species, KDR adjusts the speed and amplitude of the light-induced voltage responses [10,11,13].

The role of the transient Kv conductance, KA, is more difficult to assess. KA conductance at the dark resting potential was small (< 0.1 nS) and computer simulations demonstrated that KA had no significant role in prolonged light responses. Because of its rapid inactivation, even a 10-fold simulated increase in the KA conductance or various manipulations of voltage-dependent properties of KA had no significant effect on the light response (Figure 10). An increase in the KA current during the initial voltage transient was observed when the dark resting potential was set below the experimentally determined values. However, the physiological relevance of this finding is likely to be very small because the membrane voltage is rarely below the dark resting potential during the light stimuli. For high intensity light stimuli, the cation influx through the light-sensitive channels may induce exchanger and pump activity, which can lead to a brief hyperpolarization below the resting potential [49]. It is possible that some of the cells *in vivo* could have more negative resting potentials where KA channels could be more effectively activated. However, no systematic variation of the resting potential was found during this work, neither has this been reported in earlier studies [27].

The article "Cellular elements for seeing in the dark: voltage-dependent conductances in cockroach photoreceptors" was published in 2012. Journal: BMC Neurosci.

Besides the inter-species differences in Dipteran photoreceptor Kv channels [10], Kv channel expression can vary within the same species between photoreceptors with different functional and structural properties. In *Drosophila*, blue- and UV-sensitive photoreceptors with longer axons express larger transient Kv conductances than green-sensitive cells with short axons [50]. The transient conductance (as opposed to the alternative sustained DR type) has been suggested to decrease the attenuation of the voltage signals during propagation to the 2^nd^ order cells. Since cockroach photoreceptors have exceptionally long axons reaching over 1 mm [51], KA could serve a similar function.

Previous studies [27] and the data presented here (Figure 5A&C) indicate that a fraction of cockroach photoreceptors exhibit a particular strongly-adapting phenotype, characterized by higher KA conductance and smaller whole-cell capacitance than photoreceptors on average. *In vivo* intracellular recordings with sharp electrodes have earlier demonstrated the presence of action potential-like signals in the photoreceptor axons [26] and simulations of spiking hyper-adapting photoreceptors have shown that such combination efficiently encodes transient light intensity changes [27]. Generally, A-type Kv conductances regulate several aspects in spiking neurons [32,33,52]. We therefore hypothesize that the KA conductance could be important in tuning the transient responses in a sub-population of photoreceptors, related to signalling with either transient graded potentials or spikes in the axons. However, good quality intracellular recordings from the thin axons, 0.5 - 1 μm in diameter are lacking at present.

The functional role of the hyperpolarization activated IR current (Figure 7) is enigmatic, because its activation range is well below physiological signalling range. It could be related to transient hyperpolarization of the membrane after strong light stimulation [53]. Although a detailed study of its possible physiological function is beyond the scope of this paper, our results show that it is not carried by potassium and that substitution experiments are in accordance to its being a chloride conductance. These findings resemble a chloride current mediated by the CLC-2 channels [54], which have also been reported in the *Drosophila* photoreceptors [55].

The article "Cellular elements for seeing in the dark: voltage-dependent conductances in cockroach photoreceptors" was published in 2012. Journal: BMC Neurosci.

## Conclusions

In conclusion, we have characterized three types of voltage-dependent conductances in the cockroach photoreceptors, two Kv and one (putative) chloride conductance. The Kv-conductance composition does not conform to the previously formulated hypothesis of the roles of KDR and KA types of Kv channels in the insect photoreceptors of varying visual ecology. This earlier hypothesis was based on the studies of Dipteran flies and a more comprehensive comparative study should be conducted spanning all major insect groups. Results of such work would complement our current understanding on the different roles that Kv channels may have in photoreceptor signalling or in graded voltage signalling in general.

## Appendix

### Mathematical model of the cockroach photoreceptor

#### Glossary: model variables and parameters

*V*: membrane voltage (volts); *I*_light, KDR, KA, leak_: light-induced, KDR, KA or leak current (amperes); *C*: membrane capacitance (farads); *t*: time (seconds); *g*_light, leak_: light-dependent- or leak conductance (siemens); *G*_KDR, KA_: maximum conductance of KDR or KA (siemens); *E*_light, K_: reversal potential of light-induced or potassium current (volts); *KDR*_act_, *KA*_act_: activation parameter for KDR or KA (unitless); *KA*_inact_: inactivation parameter for KA (unitless); *τ*_Xact_, *τ*_Xinact_: activation or inactivation time constant for X (seconds).

An isopotential Hodgkin-Huxley-like model of the photoreceptor soma was constructed in Matlab programming environment (Mathworks, USA), using the measured passive, light- and voltage-dependent properties. Since we simulated the photoreceptor depolarizations arising from the light stimulation, the hyperpolarization-activated IR current was not included in the model.

#### Passive properties

The experimentally derived average whole-cell capacitance of *C* = 380 pF was used in the simulations. A passive leak conductance *g*_leak_, with reversal potential *E*_leak_ = 0 mV, was added in the model to give a resting potential of -60 mV in simulations to match the experimental conditions. The value for *g*_leak_ was calculated to give a zero net current at the resting potential. With standard Kv conductances and resting potential of -60 mV, the *g*_leak_ was 0.9 nS and resulted in a whole-cell resistance of 136 MΩ at rest and 940 MΩ at -84 mV, where the experimental input resistances were measured with the voltage clamp.

The article "Cellular elements for seeing in the dark: voltage-dependent conductances in cockroach photoreceptors" was published in 2012. Journal: BMC Neurosci.

#### Light-dependent conductance

The light-dependent conductance, *g*_light_(t), caused by light stimulation, was determined in voltage clamp. A 10 s long waveform taken from the van Hateren naturalistic stimulus database [28] was used to control the intensity of a green LED (Figure 1D bottom trace). Light-induced currents (LIC, Figure 1D) were recorded from the photoreceptors clamped to a holding potential of -74 mV in whole-cell mode. Light-dependent conductances were calculated by dividing the LIC recorded at -74 mV by the driving force of -84 mV, assuming a reversal potential of *E*_light_ = +10 mV (determined in a separate set of experiments with identical solutions).

#### Voltage-dependent properties

The voltage-dependent potassium conductances KDR and KA were incorporated in the model. The inward current was not included, since we modelled only voltages where the inward current is inactive. We used the experimentally determined potassium reversal potential of *E*_K_ = -68 mV for both the KDR and KA (Figure 3). Parameters for the voltage-dependent properties of KDR and KA are listed in Table 1. Maximum KDR conductance in the model was 78 nS, which corresponds to the mean value in the experiments. 60 nS maximum conductance value was used for the KA, which matched the value of the representative cell that was used in the model validation (Figures 8, 2D-F). KA maximum conductance was varied in the simulations without significant effect on the voltage responses, which makes this parameter non-critical (Figure 10B).

**Table 1:** Parameters for Kv conductances in the model

	**Steady-state conductance (mean ± SD)**				**Time constant (mean ± SE)**			
	***g***_***max***_**(nS)**	***V***_**50**_**(mV)**	***slope*(mV)**	***P***	**α(s**^**-1**^**)**	***slope*(V**^**-1**^**)**	**β(s**^**-1**^**)**	***τ***_***o***_**(ms)**
KDR (n = 6)	78 ± 22	-31 ± 9	12.0 ± 2.0	1	4 ± 1	43 ± 6	156 ± 53	1 ± 2
KA act. (n = 5)	36 ± 29	-43 ± 4	8.4 ± 1.6	2	*	*	*	*
KA inact. (n = 4)	-	-85 ± 1	-11.3 ± 2.9	1	341 ± 101	-44 ± 4	0.21 ± 0.07	0 ± 2

*) KA activation time constant was fixed at 1.5 ms.

*g*_*max*_ = maximum conductance, *V*_50_ = half activation/inactivation voltage, *slope* = slope factors for the steady-state parameters (Eq. 2) or time constant (Eq. 3), *P* = order for the steady-state parameter (Eq.2), α and β = activation and deactivation rates for Eq. 3, *τ*_*0*_ = offset for bell function (Eq. 3).

#### Hodgkin-Huxley-like equations

The model followed modified Hodgkin-Huxley formalism [56] where the membrane voltage *V* and activation/inactivation properties of the voltage-dependent conductances KDR and KA are described with a group of nonlinear ordinary differential equations (Eq. 1).

(1) $$\left\{ \begin{array}{l} \frac{dV}{dt}=-\left(I_{\text{LIGHT}}+I_{\text{KDR}}+I_{\text{KA}}+I_{\text{LEAK}}\right)\cdot \frac{1}{C}\\ =-\left(g_{\text{LIGHT}}\left(t\right)\left(V-E_{\text{LIGHT}}\right)+G_{\text{KDR}}KDR_{\text{act}}\left(V-E_{K}\right)+G_{\text{KA}}{\left(KA_{\text{act}}\right)}^{2}KA_{\text{inact}}\left(V-E_{K}\right)+g_{\text{LEAK}}V\right)\cdot \frac{1}{C}\\ \frac{dKDR_{\text{act}}}{dt}=\frac{KDR_{\text{s-s act}}\left(V\right)-KDR_{\text{act}}}{\tau_{\text{KDR act}}\left(V\right)}\\ \frac{dKA_{\text{act}}}{dt}=\frac{KA_{\text{s-s act}}\left(V\right)-KA_{\text{act}}}{\tau_{\text{KA act}}}\\ \frac{dKA_{\text{inact}}}{dt}=\frac{KA_{\text{s-s inact}}\left(V\right)-KA_{\text{inact}}}{\tau_{\text{KA inact}}\left(V\right)} \end{array}\right.$$

The non-inactivating KDR conductance was modelled with a single activation parameter (*KDR*_act_), whereas the inactivating KA conductance had a 2^nd^ order activation (*KA*_act_) and an inactivation (*KA*_inact_) parameter. The activation/inactivation differential equations are functions of the voltage-dependent steady-state activation/inactivation parameters (Eq. 2) and the corresponding time constants. Parameters for the equations are listed in Table 1.

(2) $$Kx_{\text{s-s act/inact}}\left(V\right)={\left(1+e^{-\frac{\left(V-V_{50}\right)}{\text{slope}}}\right)}^{-P}$$

(3) $$\tau_{\text{x act/inact}}\left(V\right)=\frac{1}{\alpha e^{-\text{slope}\cdot V}+\beta e^{\text{slope}\cdot V}}+\tau_{0}$$

The model was validated by simulating the voltage clamp subtraction protocol shown in Figure 2D-F. For validation, we used the mean activation and inactivation parameters (Figure 4A-C) and the maximum conductances for the example cell shown in Figure 2D-F (52 nS for KDR and 60 nS for KA). The voltage-clamp subtraction protocol was simulated by setting the Hodgkin-Huxley differential equation *dV*/*dt* to zero and solving the net current (*I*_*tot*_ = *I*_*KDR*_ + *I*_*KA*_ + *I*_*LEAK*_) with the voltage clamp protocol *V*(*t*) (Figure 8).

The article "Cellular elements for seeing in the dark: voltage-dependent conductances in cockroach photoreceptors" was published in 2012. Journal: BMC Neurosci.

Light responses were simulated using light-dependent conductances *g*_light_(*t*). Solving the differential equation group with the Matlab ode solver *ode23s* gave the photoreceptor voltage and activation/inactivation parameters for the conductances, which were then used to calculate the corresponding currents.

Matlab code for the simulations is available from the authors upon request.

## Competing interests

The authors declare that they have no competing interests.

## Authors’ contributions

IS analyzed the data, performed the simulations and drafted the manuscript. EI, RF, SK and YK performed experiments, analyzed the data and drafted the manuscript. MV and MW coordinated the study and drafted the manuscript. All authors read and approved the final manuscript.
